# Software Defect Prediction for Healthcare Big Data: An Empirical Evaluation of Machine Learning Techniques

**DOI:** 10.1155/2021/8899263

**Published:** 2021-03-15

**Authors:** Bilal Khan, Rashid Naseem, Muhammad Arif Shah, Karzan Wakil, Atif Khan, M. Irfan Uddin, Marwan Mahmoud

**Affiliations:** ^1^Department of Computer Science, City University of Science and Information Technology, Peshawar 25000, Pakistan; ^2^Department of IT and Computer Science, Pak-Austria Fachhochschule Institute of Applied Sciences and Technology, Haripur, Pakistan; ^3^Research Center, Sulaimani Polytechnic University, Sulimani 46001, Kurdistan Region, Iraq; ^4^Department of Computer Science, Islamia College, Peshawar 2500, Pakistan; ^5^Institute of Computing Kohat University of Science and Technology, Kohat, Pakistan; ^6^Faculty of Applied Studies, King Abdulaziz University, Jeddah, Saudi Arabia

## Abstract

Software defect prediction (SDP) in the initial period of the software development life cycle (SDLC) remains a critical and important assignment. SDP is essentially studied during few last decades as it leads to assure the quality of software systems. The quick forecast of defective or imperfect artifacts in software development may serve the development team to use the existing assets competently and more effectively to provide extraordinary software products in the given or narrow time. Previously, several canvassers have industrialized models for defect prediction utilizing machine learning (ML) and statistical techniques. ML methods are considered as an operative and operational approach to pinpoint the defective modules, in which moving parts through mining concealed patterns amid software metrics (attributes). ML techniques are also utilized by several researchers on healthcare datasets. This study utilizes different ML techniques software defect prediction using seven broadly used datasets. The ML techniques include the multilayer perceptron (MLP), support vector machine (SVM), decision tree (J48), radial basis function (RBF), random forest (RF), hidden Markov model (HMM), credal decision tree (CDT), *K*-nearest neighbor (KNN), average one dependency estimator (A1DE), and Naïve Bayes (NB). The performance of each technique is evaluated using different measures, for instance, relative absolute error (RAE), mean absolute error (MAE), root mean squared error (RMSE), root relative squared error (RRSE), recall, and accuracy. The inclusive outcome shows the best performance of RF with 88.32% average accuracy and 2.96 rank value, second-best performance is achieved by SVM with 87.99% average accuracy and 3.83 rank values. Moreover, CDT also shows 87.88% average accuracy and 3.62 rank values, placed on the third position. The comprehensive outcomes of research can be utilized as a reference point for new research in the SDP domain, and therefore, any assertion concerning the enhancement in prediction over any new technique or model can be benchmarked and proved.

## 1. Introduction

Software engineering (SE) is a discipline that is worrisome with all qualities of software development from the beginning of software specification over to keeping up to the software maintenance after it has gone into practice [1]. In the domain of SE, software defect prediction (SDP) is the utmost significant and dynamic research zone that assumes a significant job in the software quality assurance (SQA) [2, 3]. The rising convolutions as well dependencies of software systems have expanded the difficulty to deliver software with minimal effort, high caliber, and maintainability as well increase the chances of making software defects (SDs) [4, 5]. SD is a flaw or insufficiency in a software system that roots the development of a spontaneous result. An SD can moreover be the situation when the last software product does not meet the client's desire or client prerequisite [6]. SD's can cause the diminution of the software product quality and increase the development cost.

SDP is a momentous commotion to assure the substances of a software system that leads to adequate development cost and recover the quality by identifying defect-prone instances before testing [4]. It moreover embraces categorizing software components in different varieties of a software system that constructs the testing progression supplementary by concentrating on testing as well as evaluating the components classified as defective [7]. Defects adversely affect software reliability and quality [8].

SDP in the primary period of the software development life cycle (SDLC) is measured as an utmost thought-provoking aspect of SQA [9]. In SE, bug fixing and testing are very costly which also require a massive amount of resources. Forecasting the software defects in software development has been observed by numerous studies in the last decades. Amid all these studies, machine learning (ML) techniques are considered as the best approach toward SDPs [7, 10, 11].

Keeping the above issue related to SDP, various researchers evaluated and built SDP models utilizing diverse classification techniques. Still, it is quite challenging to sort any broad-spectrum preparation to inaugurate the usability of these techniques. Inclusively, it was originated that notwithstanding some dissimilarities in the studies, no particular SDP technique delivers higher to the other techniques diagonally different datasets. The researchers have utilized different evaluation measures to assess the projected models to find the best model for SDP [12, 13].

However, this study focuses on the empirical analysis of ten ML techniques amid which some are proposes as new solutions for SDP. ML techniques include the multilayer perceptron (MLP), radial basis function (RBF), support vector machine (SVM), decision tree (J48), random forest (RF), hidden Markov model (HMM), credal decision tree (CDT), *K* -nearest neighbor (KNN), average one dependency estimator (A1DE), and Naïve Bayes (NB) for SDP. Amid all these techniques, HMM and A1DE are proposed aimed for the first time for SDP. These techniques are employed on seven different datasets including AR1, AR3, CM1, JM1, KC2, KC3, and MC1. All the experiments are validated using relative absolute error (RAE), mean absolute error (MAE), root relative squared error (RRSE), root mean squared error (RMSE), recall, and accuracy.

Following is a list of the contributions of this research:

1. To benchmark ten different ML techniques (MLP, J48, SVM, RF, RBF, HMM, CDT, A1DE, KNN, and NB) for SDP
2. To demeanor a series of try-outs on different datasets such as AR1, AR3, CM1, JM1, KC2, KC3, and MC1
3. To reveal insight into the experimental outcomes, evaluation is accomplished using MAE, RAE, RMSE, RRSE, recall, and accuracy
4. To show that experimental outcomes are significantly different and comparable with verifying the best results, Friedman two-way examination of difference by ranks is performed

Hereinafter, Section 2 presents the literature survey, Section 3 comprises the methodology and techniques, while experimental outcomes are discussed in Sections 4, and Section 5 covers the inclusive conclusion.

## 2. Literature Survey

This section delivers an ephemeral study about existing techniques in the field of SDP. Several researchers have employed ML techniques for SDP at the initial phase of software development. Several particular studies converse here. Czibula et al. [11] presented a model grounded on relational association discovery (RAD) for SDP. They apply all investigations on NASA dataset including KC1, KC3, MC2, MW1, JM1, PC3, PC4, PC1, PC2, and CM1. To assess the model as compared to other models, use accuracy, precision, specificity, probability of detection (PD), and area under cover (ROC) assessment measure. The acquired outcomes present that RAD perform well rather than other employed techniques.

A framework for SDP named the Defect Prediction through Convolutional Neural Network (DP-CNN) has been recommended by Li et al. [14]. The authors evaluated the DP-CNN on seven different open source projects such as Camel, jEdit, Lucene, Xalam, Xerces, Synapse, and Poi in terms of *F*-measure in defect predictions. Overall outcomes illustrate that on average, the DP-CNN enhanced the up-to-the-minute technique by 12%.

Jacob and Raju [15] introduced a hybrid feature selection (HFS) method for SDP. They also perform their analysis on NASA datasets including PC1, PC2, PC3, PC4, CM1, JM1, KC3, and MW1. The outcomes of HFS are benchmarked with Naïve Bayes (NB), neural networks (NN), RF, random tree (RT), and J48. Benchmarking is carried out using accuracy, specificity, sensitivity, and Matthew's correlation coefficient (MCC). The analyzed outcome shows that HFS outperform while improving classification accuracy from 82% to 98%.

Bashir et al. [16] presented a joined framework to improve the SDP model using Ranker feature selection (RFS), data sampling (DS), and iterative partition filter (IPF) techniques to conquest class imbalance, noisy correspondingly, and high dimensionality. Seven ML techniques including NB, RF, KNN, MLP, SVM, J48, and decision stump are employed on CM1, JM1, KC2, MC1, PC1, and PC5 datasets for evaluations. The outcomes are carried out utilizing receiver operating characteristic (ROC) performance evaluation. Overall experimental outcomes of the proposed model outperformed other models.

A new approach for SDP utilizing a hybridized gradual relational association (HyGRAR) and artificial neural network (ANN) to classify the defective and nondefective objects is projected in [7]. Experiments were achieved based on ten different open source datasets such as Tomcat 6.0, Anr 1.7, jEdit 4.0, jEdit 4.2, jEdit 4.3, AR1, AR3, AR4, AR5, and AR6. For module evaluation, accuracy, sensitivity, specificity, and precision measures were utilized. The author concluded that HyGRAR achieved better outcomes as compared to most of the foregoing projected approaches.

Alsaeedi and Khan [8] performed the comparison on supervised learning techniques including bagging, SVM, decision tree (DT), and RF and ensemble classifiers on different NASA datasets such as CM1, MC1, MC2, PC1, PC3, PC4, PC5, KC2, KC3, and JM1. The basic learning and ensemble classifiers are evaluated using *G*-measure, specificity, F-score, recall, precision, and accuracy. The experimental results conducted show that RF, AdaBoost with RF, and DS with bagging outperform than other employed techniques.

The author in [9] performed comparative exploration of several ML techniques for SDP on twelve NASA datasets such as MW1, CM1, JM1, PC1, PC2, PC3, PC4, PC5, KC1, KC3, MC1, and MC2, while the classification techniques include one rule (OneR), NB, MLP, DT, RBF, kStar (K^∗^), SVM, KNN, PART, and RF. The performance of each technique is assessed using MCC, ROC area, recall, precision, *F*-measure, and accuracy.

Malhotra and Kamal [6] evaluated the efficiency of ML classifiers for SDP on twelve excessive datasets taken from the NASA repository by employing sampling approaches and cost-sensitive classifiers. They examine five prevailing methods including J48, RF, NB, AdaBoost, and bagging, as well as suggest the SPIDER3 method for SDP. They have compared the performance based on accuracy, sensitivity, specificity, and precision.

Manjula and Florence [17] developed a hybrid model of the genetic algorithm (GA) and the deep neural network (DNN). GA is utilized for feature optimization while DNN is for classification. The enactment of the projected technique is benchmarked with NB, RF, DT, Immunos, ANN-artificial bee colony (ABC), SVM, majority vote, AntMiner+, and KNN. All the performances are carried out on a dataset that includes KC1, KC2, CM1, PC1, and JM1 and assessed via recall, F-score, sensitivity, precision, specificity, and accuracy. The tentative results show that the recommended technique beats other techniques in terms of achieving better accuracy.

Researchers have used various techniques to incredulous the boundaries of SDP on a variety of datasets. In each study, different evaluation measures are accomplished to evaluate and benchmark the proposed techniques. The overall summary of the literature discussed above is listed in Table 1, where the first column represents the authors who conducted research studies utilizing various ML techniques. The second column of the table shows techniques utilized by an individual study, while the third and fourth columns represent dataset and evaluation measures utilized in different studies. As shown in Table 1, each study has used different evaluation measures to achieve higher accuracy, but none affects decreasing error rate which is a significant feature.

Moreover, the ML techniques are also utilized by many researchers in healthcare engineering and the development of medical data analyzing software [1]. Khan et al. [2] utilized machine learning techniques for the prophecy of chronic kidney disease (CKD) to suggest the best model of early prediction of CKD. The study of Makumba et al. [3] on heart disease prediction using data mining (DM)/ML techniques can also be the baseline for new researchers. They have employed the DM/ML techniques on heart disease datasets. Hence, many researchers have utilized ML techniques on different healthcare datasets for early prediction of disease. However, the most important task is that when they propose an optimal solution for any kind of disease, they also have to give the assurance for the quality of software that will be developed using their optimal solution. To ensure this, we have to predict the defect that may occur in the software which leads towards decreasing the quality of the software system. Those are the reasons behind this research study.

## 3. Methodology and Techniques

This study objects to present the performance analysis of ML techniques for SDP on various datasets including AR1, AR3, CM1, JM1, KC2, KC3, and MC1. All these datasets can be found on the UCI ML repository (https://archive.ics.uci.edu/). The experimentation is performed using the open source ML and DM tool Weka version 3.9 (https://machinelearningmastery.com/use-ensemble-machine-learning-algorithms-weka/). As per the information presented in Table 1, AR1 and AR3 are reported in the literature single time; as shown in Figure 1, CM1 and JM1 reported 6 times, KC2 and MC1 reported 1 time, while KC3 reported 4 times. Each dataset is consisting of some attributes along with known output class. Respectively, datasets contain numerical data, while the total numbers of attributes and instances are different as presented in Table 2. In Table 2, the first column shows the datasets and second and third columns present number of metrics (attributes) and several cases (instances) correspondingly. The fourth and fifth columns represent the number of defective modules and the number of nondefective modules correspondingly, while the last column shows the type of data in each dataset. However, Table 3 shows the list of all attributes (software metrics) according to each dataset utilized in this research. The experimental setup for SDP is shown in Figure 2, which explains how each task is performed in this research. After training the datasets, the preprocessing step is taken only on the class attribute of each dataset that is solitary to change the type of data from numerical to categorical due to some of the ML techniques unable to work on numerical type class attributes. After all, when ML techniques apply to each dataset, the outcome is assessed using different assessment measures to show the better performance of an individual technique. Therefore, six assessment measure named MAE [13, 18, 19], RMSE [8, 20, 21], RAE [16, 22, 23], RRSE [22, 24], recall [9, 10, 25], and accuracy [26–28] are utilized to evaluate the performance of ML techniques on SDP datasets. We have used error-based assessment measures which are not reported in the literature, while recall and accuracy have been used 3 and 7 times, respectively (Figure 3).

Table 4 shows the calculation mechanism and a description of each evaluation measure. The second column of Table 4 shows the list of evaluation measures, while the third column represents the equation of each measure, where, |*y*_*i*_ − *y*| is the absolute error, *n* is the number of errors, *T*_*j*_ is the goal value for record *ji*, *P*_*ij*_ is the prediction value by the particular technique *I* for record *j* (beyond *n* records), TP is the quantity of true-positive classification, FN is the amount of false-negative classification, TN is the amount of true-negative classification, and FP is the quantity of false-positive classifications.

## 4. Techniques Employed

ML techniques are currently extensively used to excerpt significant knowledge commencing massive volumes of data in diverse areas. ML applications embrace numerous real-world situations such as cyber-security, bioinformatics, detecting communities in social networks, and software process enhancement to harvest high-quality software systems [7]. ML-based solutions for SDP have also been investigated [6, 10, 29]. From which, we have selected the top seven techniques as reported in Table 1, and the count of each technique is given in Figure 4. RBF is selected randomly, while the other two, i.e., HMM and A1DE, are new explorations for SDP. All of the ten selected techniques are briefly discussed in the following subsections.

### 4.1. Support Vector Machine

SVM has numerous uses in the field of classification, biophotonics, and pattern recognition [8, 25]. First, it was developed for binary classification; however, it can also be used for multiple classes [30]. In binary classification, the core impartial of SVM is to describe a line among classes of data to exploit the remoteness of edge line from data points lying neighboring to it. In that case, if data are linearly inseparable, a mathematical function is utilized to transmute the data to a higher-attribute space, so that it may become linear divisible in the new space. The function used is called kernel function, and the equation of a linear SVM can be written as

(1) $$\begin{array}{c} f\left(x\right)=\;\sum_{i=0}^{N}\alpha_{i}y_{i}x_{i}^{T}.x+\beta_{0}, \end{array}$$

where *x*_*i*_ is the prompt with label *y*_*i*_, *α* is the Lagrange multiplier, and *β*_0_ is the partiality, while *N* signifies the number of support vectors. For nonlinearly divisible issue, the overhead equation can be improved for kernel SVM as

(2) $$\begin{array}{c} f\left(x\right)=\;\sum_{i=0}^{N}\alpha_{i}y_{i}K\left(x_{i}.x\right).x+\beta_{0}, \end{array}$$

where *K*(*x*_*i*_.*x*) is the kernel function.

### 4.2. Decision Tree (J48)

This is the basic C4.5 decision tree (DT) used for classification problems [26]. It is the deviation of information gain (IG), usually utilized to stun the result of unfairness. An attribute with a maximum gain ration is nominated in direction to shape a tree as a splitting attribute. Gain ratio- (GR-) based DT performs well as compared to IG [31], in terms of accuracy. GR is defined as

(3) $$\begin{array}{c} {\text{Gain}}_{\text{ratio }\left(D.A\right)}=\;\frac{\text{Entropy}\left(D\right)\sum_{j=1}^{l}\left(P_{j}.\text{entropy}\left(P_{j}\right)\right)}{{\text{Spliting}}_{\text{info}}}. \end{array}$$

### 4.3. Random Forest

It produces a set of techniques that involve constructing an ensemble or termed as a forest of decision trees from a randomized variation of tree induction techniques [32]. RF works by forming a mass of decision trees at the training period and harvesting the class in the approach of the class output by a single tree [33]. It is deliberated as one of the utmost techniques which is extremely proficient for both classification and regression problems.

### 4.4. Multilayer Perceptron

MLPs are deliberated as the utmost momentous classes of the neural network including an input layer, output layer, and least one hidden layer [34–36]. The techniques behind the neural network are that when data are accessible as the input layer, the network neurons start calculation in the sequential layer until an output value is gained at each of the output neurons. A threshold node is moreover added in the input layer which identifies the weight function. The resultant calculations are used to gain the activity of the neurons by smearing a sigmoid activation function that can be defined as

(4) $$\begin{array}{c} P_{j}=\;\sum_{i=1}^{n}w_{j,i}x_{i}+\theta_{j},m_{j}=\;f_{j}\left(p_{j}\right), \end{array}$$

where *P*_*j*_ is the linear combination of inputs *x*_1_, *x*_2_,…, *x*_*n*_, *θ*_*j*_ is the threshold, *w*_*j*,*i*_ is the connection weight between *x*_*i*_ and neuron *j*, *f*_*j*_ is the activation function of the *j*^th^ neuron, and *m*_*j*_ is the output. A sigmoid function is a mutual choice of activation function that can be described as

(5) $$\begin{array}{c} f\left(t\right)=\;\frac{1}{1+\;e^{-t}}. \end{array}$$

### 4.5. Radial Basis Function

It is also a neural network model that needs a very few computational time for training a network [37, 38]. Likewise, MLP also contains input, hidden, and output layers. The input variables in the input layer permit straight to the hidden layer deprived of weights. The transfer functions of the hidden knobs are RBFs, which factors are elevated throughout the training. The process of appropriating RBFs to data, for function of rough calculation, is thoroughly associated with space-weighted regression.

### 4.6. Hidden Markov Model

HMM is a probabilistic or [39] a statistical Markov model where the scheme being modeled is probable to be a Markov procedure using unobservable states or hidden statuses. It can be epitomized as the gentlest dynamic Bayesian network. It is reliant on splitting large data into the smallest sequences of data using a fewer sensitive pairwise sequence comparison method [40]. This model can be reflected in the generality of a combination model where the hidden variables that control the combination section to be nominated for every statement are connected through a Markov process moderately than liberated from each other. HMMs are particularly identified for their use in reinforcement learning and chronological pattern recognition such as speech, handwriting, part-of-speech tagging, gesture recognition, partial discharges, musical score following, and bioinformatics [39, 41].

### 4.7. Credal Decision Tree

Credal decision trees (CDTs) are algorithms to design classifiers grounded on inexact possibilities and improbability measures [42]. Throughout the creation procedure of a CDT, to sidestep producing a very problematical decision tree, a new standard was presented: stay once the total improbability rises due to splitting of the decision tree. The function utilized in the total hesitation dimension can be fleetingly articulated as [43, 44]

(6) $$\begin{array}{c} \text{TU }\left(\xi \right)=\text{IG}\left(\xi \right)+\text{GG}\left(\xi \right), \end{array}$$

where *ξ* is a Credal fixed on frame *X*, TU is the value of total hesitation, IG represents a common function of nonspecificity on the resultant Credal set, and GG is a common function of arbitrariness for a Credal set.

### 4.8. Average One Dependency Estimator

A1DE is a probabilistic technique used for mostly classification problems. It succeeds extremely precise classification by averaging inclusive of a minor space of different NB-like models that have punier independence suppositions than NB. A1DE was designed to address the attribute-independence issues of a popular NB technique. It was designed to address the attribute-independence issues of the prevalent naive Bayes classifier. A1DE pursues to estimate the possibility of every class *y* assumed a quantified set of features *x*_1_*, x*_2_,…, *x*_*n*_,*P*(*y|x*_1_,…, *x*_*n*_) [45]. This can be calculated as

(7) P^y|x1,x2,…,xn= ∑i:1≤n∧Fxi≥mP^y,xi∏j=1nP^y,xi∑y′∈Y ∑i:1≤i≤n∧Fxi≥mP^y′,xi∏j=1nP^xi|y′,xi,

where $\hat{P}\left(.\right)$ represents an assessment of *P*(.), *F*(.) is the frequency through which the influences seem in the trial data, and *m* is a user quantified least frequency by which a term essentially seems in direction to be utilized in outer summation. Currently, *m* is the habitually set at 1.

### 4.9. Naïve Bayes

NB is a kinfolk of modest probabilistic technique grounded on Bayes theorem with unconventionality suppositions amid the predictors [46, 47]. The NB model is precise simple to construct and can be executed for any dataset containing a large amount of data. The posterior probability, *P*(*c|x*), is taken from *P*(*c*), *P*(*x*), and *P*(*x|c*). The consequence of the value of a forecaster (*x*) on assumed class (*c*) is independent of the value of other forecasters.

(8) $$\begin{array}{c} P\left(c|x\right)=\;\frac{P\left(x|c\right)P\left(c\right)}{P\left(x\right)}\text{ or}\\ \text{Posterior}=\;\frac{\text{Prior}{}^{*}\text{likelihood}}{\text{Evidence}}. \end{array}$$

### 4.10. *K*-Nearest Neighbor

KNN is a supervised learning technique where the preparation of features attributes to forecast the class of new test data. KNN classifies first-hand data grounded on the least distance from the new data to the *K*-nearest neighbors [48, 49]. The nearest distance can be found using different distance functions such as Euclidean distance (ED), Manhattan distance (MD), and Minkowski distance (MkD). Here, in this study, ED is used that can be formulated as

(9) $$\begin{array}{c} d\left(X,\;Y\right)=\;\sqrt{\sum_{i=1}^{k}{\left(x_{i}-y_{i}\right)}^{2}}, \end{array}$$

where *X* = (*x*_1_, *x*_2_,…, *x*_*n*_) and *Y* = (*y*_1_, *y*_2_,…, *y*_3_).

## 5. Experimental Results

### 5.1. Results and Analysis

This section provides an experimental study for SDP employing ten ML techniques using a standard approach of the 10-fold cross-validation process for assessment [34]. This process splits the complete data into ten subgroups of equal sizes; one subgroup is used for testing, whereas the rest of the subgroups are used for training. This process is continuing until each subgroup has been used for testing.

In this work, we considered seven different software defect datasets named AR1, AR3, CM1, JM1, KC2, KC3, and MC1. Using these datasets, we apply a software defect prediction system where the performance of all employed ML techniques is compared with each other based on correctly and incorrectly classified instances, true-positive and false-positive rates, MAE, RAE, RMSE, RRSE, recall, and accuracy.  Table 5 presents the benchmark analysis of correctly classified instances (CCI), while Table 6 presents the benchmark analysis of incorrectly classified instances (ICI) using ML techniques. In both tables, the first column represents techniques employed, while the rest of the columns show details of each dataset concerning CCI and ICI.  Figure 5 shows the inclusive performance CCI and ICI evaluation of each employed ML technique.

Table 7 illustrates the true-positive rate (TPR) and false-positive rate (FPR) of each technique on different hired datasets. TPR reveals the probability of the positive modules correctly classified, while FPR defines the probability of the negative modules incorrectly classified as the positive modules [5]. The first column of the table shows the list of datasets used, while the second column represents the TPR and FPR on the respective dataset. Apart from this, each row represents the achieved TPR and FPR concerning the individual dataset.

Tables 8 and 9 show the outcomes of absolute errors that are MAE and RAE, respectively. In each table, the first column represents the list of techniques, while the rest of the columns represent the error rate of each dataset concerning techniques employed. As shown in Table 8, while calculating MAE, SVM performs well in reducing the error rate as associated to other utilized techniques. SVM produces better results on five datasets, while MLP and NB produce better results only on two datasets. In the case of calculating RAE, SVM creates better results utilizing four datasets, while A1DE and NB do the same only for one dataset individually. This determines to calculate the absolute error, and SVM outperforms other techniques.

However, Tables 10 and 11 present the outcomes of each squared error that are RMSE and RRSE individually. Here, the outcomes of squared error are different than outcomes of absolute error. While calculating RMSE or RRSE in both cases, RF produces better results for three datasets that are JM1, KC3, and MC1, RBF for two datasets that are CM1 and KC2, whereas MLP and CDT for only one dataset separately that are AR3 and AR1, respectively. Although, this analysis shows the best performance of RF as compared to other employed ML techniques.

Table 12 shows the outcomes achieved using recall assessment measures. In this table, the first row represents the list of datasets, while the first column represents the list of employed techniques. The rest of the rows concerning individual techniques shows the outcomes utilizing each dataset. This table shows that calculating recall using the AR1 dataset, HMM, and CDT performs well and produces the same results of 0.926. Proceeding utilizing AR3 and KC2 datasets, MLP outperforms other techniques generating 0.937 and 0.847 correspondingly, while on CM1 and AR1 datasets, HMM and on KC3 and AR1 datasets CDT performs well while producing 0.926 and 0.902 results. Moreover, on MC1 and JM1 datasets, the results of RF are better as compared to other techniques that are 0.827 and 0.995 accordingly; while, on the KC3 dataset, SVM performance is better, that is, 0.82.  Figure 6 presents the overall recall performance of ML techniques for datasets. It can be concluded that RF, MLP, HMM, and CDT have better performed in terms of recall.

Table 13 shows the accuracy performance of each employed technique using different datasets. In this table, the first column represents the list of techniques, whereas the first row represents the list of datasets. The rest of the columns and rows show the outcome of each technique utilizing every dataset. Amid all the outcomes, the better performance of each technique under the individual dataset is listed in bold as shown in Table 13. This analysis shows that HMM produces better accuracy on three datasets, namely, AR1, AR3, and CM1, and outcomes are 92.562%, 97.3016%, and 90.1606%, respectively. RF harvests better accuracy on JM1 and near to best on MC1, that is, 82.6644% and 99.4824%, while SVM and MLP create better accuracy for KC3 and KC2, that is, 81.9588% and 84.6743%, respectively. Utilizing the MC1 dataset, A1DE outperforms other techniques achieving the accuracy of 99.4929%. The clinched performance of all techniques on individual datasets is presented in Figure 7.

Our outcomes suggest that there is uncertainty in the ML techniques. No individual technique performs well on every dataset. Different assessment measures are utilized to test the performance of each ML techniques on every dataset.  Table 14 also presents the ranking of each technique, where we can see that HMM produces better results on 3 datasets; this number is maximum from the better results produced by any other techniques. However, on average, RF produces better results (average rank = 2.96), and the KNN produced poor results (average rank = 6.68). This is due to RF produces the forest with several trees [33, 50]. Overall, the more trees in the forest, the more forceful the forest resembles. Likewise in the RF classifier, the large amount of trees in the forest causes to give higher accuracy results [51, 52].

To get insight into the number, Table 13 shows the overall decision for SDP utilizing ML techniques on AR1, AR3, CM1, JM1, KC2, KC3, and MC1 datasets. This table concludes that which technique performs well on an individual dataset to a specific assessment criterion.

A standard approach to benchmark the performances of classifiers is to count (*w*) the number of datasets on which an algorithm is an overall subjugator, also known as the Count of Wins test. We have used 7 datasets, and no technique has given the best results for at least 7 datasets at *α* = 0.05, according to the critical values in Table 3 of [53]. Since the Count of Wins test is also considered to be a weak testing procedure, therefore, we have a detailed matrix Table 14. As it can be observed from the very first dataset from Table 14, that is AR1, CDT outperforms other techniques in terms of increasing accuracy and reducing squared error while reducing absolute errors; MLP and SVM also perform well. On second and third datasets such as AR3 and CM1, HMM outperforms other techniques in terms of increasing accuracy; however, reducing the error rate on the AR3 dataset, MLP and A1DE produces better results, and utilizing the CM1 dataset, SVM and RBF performs well. Moreover, using JM1 and MC1, RF and KNN produce better results in terms of increasing accuracy and decreasing squared error rate, while decreasing absolute error SVM and KNN outperform well. Furthermore, on the KC2 dataset, MLP performs well in increasing accuracy, and using the KC3 dataset, SVM performs well. However, on KC2 and KC3, SVM, RF, RBF, and NB performance is better in terms of reducing error rates.

All the employed techniques perform well certain in terms of reducing error rate, while some in terms of increasing accuracy, excluding J48. J48 is an insecure technique, for data containing categorical variables with a diverse number of altitudes as we have in employed datasets, and information gain in the decision tree is unfair in service of those metrics with more levels and fairly imprecise [54]. The performance of every individual technique is different on each singular dataset, which is due to the change of population in each dataset as well as differences between the values range and a number of attributes.

### 5.2. Friedman Two-Way Analysis of Variance by Ranks

To compare all applied ML techniques on numerous datasets, we have smeared the statistical technique as defined by Sheskin [55] and García [56]. The Friedman two-way analysis of difference by ranks (Friedman) [57] is adopted with rank-order data in a hypothesis testing condition. A significant test specifies that there is a significant variance amid at least two of the techniques in the set of *k* techniques. The Friedman test checks whether the measured average ranks are significantly different from the mean rank (in our case, *R*_*j*_ = 4.54). The chi-square (*χ*^2^) distribution is used to approximate the Friedman test statistic [55]. Friedman's statistic is

(10) $$\begin{array}{c} X^{2}=63.218. \end{array}$$

To throw away the null hypothesis, the workout value must be equal to or greater than *χ*^2^, the tabled (table of the chi-square distribution) precarious chi-square value at the prespecified level of significance [55]. The number of degrees of freedom d*f* = *k* − 1. Thus, d*f* = 10 − 1 = 9. For d*f* = 9, the tabled critical *α* = 0.05 and chi-square value *χ*^2^ = 16.92. Since the computed value = 63.218 is greater than *χ*^2^_0.05_ = 16.92, the alternative hypothesis is supported at *α* = 0.05. It can be concluded that there is a significant difference among at least nine of the ten ML techniques. This result can be summarized as follows: *χ*^2^_0.05_ (9) = 63.218, *P* < 0.05.

Since the critical value is lower than *χ*^2^, we can continue with posthoc tests to spot the significant pairwise differences among all the techniques. The results are shown in Table 15, where *z* is the corresponding statistics and *P* values are for each hypothesis. *Z* is computed using the following equation:

(11) $$\begin{array}{c} z=\frac{\left(R_{i}-R_{j}\right)}{\text{SE}}, \end{array}$$

where *R*_*i*_ is the *i*^th^ technique, and the standard error is $\text{SE}=\sqrt{\left(k\left(k+1\right)\right)/6n}=0.249$. Columns 5 and 6 represent Nemenyi's and Holm's static procedure. The second last column lists the differences between the average ranks of *i*^th^ and *j*^th^ techniques. While, the last column shows the critical difference (CD), and it states that the performance of the two techniques is expressively diverse if the consistent average ranks differ by at least the CD. CD can be assessed using

(12) $$\begin{array}{c} \text{CD}=q\alpha \sqrt{\frac{k\left(k+1\right)}{6n}}, \end{array}$$

where critical values *qα* is given in (Table 5(b), Demsar 2006) [53]. The notations “>” and “<” represent whether the difference of the average rank (*R*_*i*_ − *R*_*j*_) is greater or less than the value of CD, respectively. Greater means a significant difference between two means. Here, the value of CD is 0.692.

In Table 15, the family of hypotheses is ordered by their *P* values. As can be seen, Nemenyi's procedure rejects the first 27 hypotheses, whereas Holm's procedure also rejects the next 4 hypotheses; meanwhile, the corresponding *P* values are lesser than the adjusted NM-*α*'s and Holm. Hence, we conclude that the performance of MLP and CDT is comparable, and KNN has a lower performance. Besides, the obtained value CD = 0.692 specifies that any variance amid the average ranks of two techniques that is equal to or greater than 0.692 is significant. Concerning the pairwise comparisons in Table 15, the difference between the average ranks of two techniques which are greater than CD = 0.692 is the first 32. Thus, it can be concluded that there is a momentous alteration among the average ranks of the first 32 pairs of techniques.

## 6. Threats to Validity

This section converses the effects that could anguish the validity of this research work.

### 6.1. Internal Validity

The exploration of this study is grounded on diverse very familiar valuation standards that are used in the past in various studies. Amid these standards, several are used to assess the error rate while certain used to assess the accuracy. So, the treat can be that the renewal of new valuation standards as a replacement for utilized standards may deteriorate the accuracy. Furthermore, the machine learning techniques used in this study may be replaced with other existing techniques and can be merged that can harvest enhanced outcomes than the employed techniques.

### 6.2. External Validity

We piloted investigations on various datasets. A threat to validity may arise if the projected techniques are related in the other actual data composed from the diverse software development organizations using surveys or replace these datasets with some other datasets, which may distress the outcomes while growing the error rates. Likewise, the projected technique might not be capable to harvest improved forecast in outcomes utilizing several other SDP datasets. Hence, this study concentrated on AR1, AR3, CM1, JM1, KC2, KC3, and MC1 datasets to measure the performance of the utilized techniques.

### 6.3. Construct Validity

Diverse ML techniques are benchmarked with each on various datasets on the base of several valuation standards. The assortment of techniques utilized in this study is on the canter of their progressive features over other techniques that ought to exploit by the researchers in the last decades. Though the threat can be that we put on several new techniques, at that point, it can be the probability that these new techniques can exhaust the projected techniques. Furthermore, the training and testing method is applied or we change the number of folds validation (increase or decrease) for the experimentations that can decrease the error rate. It moreover can be promising that using the newest valuation standards creates improved outcomes that can beat the current accomplished outcomes.

## 7. Conclusions

Nowadays SDP using ML techniques is dignified as one of the developing research zones. The identification of software defects at the primary phase of SDLS is a challenging task, as well it can subsidize the provision of high-quality software systems. This study focused on comparing seven famous ML techniques that are broadly used for SDP, on seven extensively used openly available datasets. The ML techniques include SVM, J48, RF, MLP, RBF, HMM, and CDT. The performance is evaluated utilizing different measures such as MAE, RAE, RMSE, RRSE, recall, and accuracy.

The experimental results have illustrated that NB and SVM produced fewer MAE and RAE, respectively. However, experimental results using RMSE, RRSE, recall, and accuracy showed that an average RF performed better. Friedman's two-way analysis of variance by ranks has performed on experimental results using accuracy. The Friedman test indicates that results are significant at *P* < 0.05. We also performed a pairwise statistical test which revealed that several pairs are significant. Moreover, a critical difference test showed that RF and KNN produced significantly different results at *P* < 0.05, where RF produced better while KNN the poorest. The outcomes obtainable in this study may be recycled as the reference point for other studies and researchers, in such a way that the outcomes of any projected technique, model, or framework can be benchmarked and simply confirmed. For future works, class imbalance matters ought to be committed to these datasets. Furthermore, to increase the enactment, ensemble learning and feature selection techniques could also be explored.

## Figures and Tables

**Figure 1:** Count of reported datasets.

**Figure 2:** Software defect prediction model.

**Figure 3:** Count of reported measures.

**Figure 4:** Count of each technique.

**Figure 5:** ML techniques performance comparison on CCI and ICI using SDP datasets.

**Figure 6:** Recall comparison of ML technique using an individual dataset.

**Figure 7:** Accuracy comparison of ML technique using an individual dataset.

**Table 1:** Summary of the literature survey.

Author	Technique/Model	Datasets	Evaluation measures
Czibula et al. [11]	RAD	MW1, JM1, PC1, PC2, PC3, PC4, KC1, KC3, MC2, and CM1	Accuracy, specificity, precision, PD, and ROC
Li et al. [14]	DP-CNN	Camel, jEdit, Lucene, Xalam, Xerces, Synapse, and Poi	*F*-measure
Jacob and Raju [15]	HFS, NB, NN, RF, RT, J48	PC1, PC2, PC3, PC4, CM1, MW1, KC3, and JM1	Specificity, sensitivity, MCC, and accuracy
Bashir et al. [16]	NB, RF, KNN, MLP, SVM, J48, and decision stump	CM1, JM1, KC2, MC1, PC1, and PC5	ROC
Miholca et al. [7]	HyGRAR	Tomcat 6.0, Anr 1.7, jEdit 4.0, AR1, jEdit 4.2, AR3, jEdit 4.3, AR5, AR4, and AR6	Accuracy, sensitivity, specificity, and precision
Alsaeedi and Khan [8]	Bagging, SVM, DT, and RF	PC1, PC3, PC4, PC5, JM1, KC2, KC3, MC1, MC2, and CM1	*G*-measure, specificity, *F*-score, recall, precision, and accuracy
Iqbal et al. [9]	OneR, NB, K^∗^, MLP, SVM, RBF, RF, KNN, DT, and PART	JM1, MW1, CM1, MC1, PC1, MC2, PC4, PC3, PC2, PC5, KC3, and KC1	MCC, ROC area, *F*-measure, recall, precision, and accuracy
Malhotra and Kamal [6]	J48, RF, NB, AdaBoost, and bagging, and SPIDER3	NASA datasets	Accuracy, sensitivity, specificity, and precision
Manjula and Florence [17]	GA, DNN, NB, RF, DT, ABC, SVM, and KNN	KC1, KC2, CM1, PC1, and JM1	Precision, sensitivity, specificity, recall, *F*-score, and accuracy

**Table 2:** Attributes, instances, defective, and nondefective modules of each utilized dataset.

S. No.	Datasets	No. of attributes	No. of instances	No. of defective modules		No. of nondefective modules		Data type
1	AR1	30	121	9	7.4%	112	(92.6%)	Numerical
2	AR3	30	63	8	12.7%	55	(87.3%)	Numerical
3	CM1	22	498	49	9.8%	449	(90.2%)	Numerical
4	JM1	22	9593	1759	18.3%	7834	(81.7%)	Numerical
5	KC2	22	522	107	20.5%	415	(79.5%)	Numerical
6	KC3	40	194	36	18.6%	158	(81.4%)	Numerical
7	MC1	40	9466	68	0.7%	9398	(99.3%)	Numerical

**Table 3:** List of attributes according to datasets.

Attributes		Datasets						
		AR1	AR3	CM1	JM1	KC2	KC3	MC1
Halstead attributes	Halstead content	✓	✓	—	✓	-	✓	✓
	Halstead difficulty	✓	✓	✓	✓	✓	✓	✓
	Halstead effort	✓	✓	✓	✓	✓	✓	✓
	Halstead error estimator	✓	✓	—	✓	-	✓	✓
	Halstead length	✓	✓	✓	✓	✓	✓	✓
	Halstead level	✓	✓	✓	✓	✓	✓	✓
	Halstead program time	✓	✓	✓	✓	✓	✓	✓
	Halstead volume	✓	✓	✓	✓	✓	✓	✓
	Number of operands	✓	✓	✓	✓	✓	✓	✓
	Number of operators	✓	✓	✓	✓	✓	✓	✓
	Number of unique operands	✓	✓	✓	✓	✓	✓	✓
	Number of unique operators	✓	✓	✓	✓	✓	✓	✓
McCabe attributes	Essential complexity	—	—	✓	✓	✓	✓	✓
	Cyclomatic complexity	✓	✓	✓	✓	✓	✓	✓
	Design complexity	✓	✓	✓	✓	✓	✓	✓
	Cyclomatic density	✓	✓	—	—	—	✓	✓
Size attributes	Number of lines	—	—	✓	-	✓	✓	✓
	LOC total	✓	✓	✓	✓	✓	✓	✓
	LOC executable	✓	✓	—	✓	—	✓	✓
	LOC comments	✓	✓	✓	✓	✓	✓	✓
	LOC code and comments	✓	✓	✓	✓	✓	✓	✓
	LOC blank	✓	✓	✓	✓	✓	✓	✓
Others attributes	Branch count	✓	✓	✓	✓	✓	✓	✓
	Condition count	✓	✓	—	—	—	✓	✓
	EDGE count	—	—	—	—	—	✓	✓
	Parameter count	✓	✓	—	—	—	✓	✓
	Modified condition count	—	—	—	—	—	✓	✓
	Multiple condition count	✓	✓	—	—	—	✓	✓
	Node count	—	—	—	—	—	✓	✓
	Design density	✓	✓	—	—	—	✓	✓
	Essential density	—	—	—	—	—	✓	✓
	Decision count	✓	✓	—	—	—	✓	✓
	Decision density	✓	✓	—	—	—	✓	-
	Call pairs	✓	✓	—	—	—	✓	✓
	Global data complexity	—	—	—	—	—	✓	✓
	Global data density	—	—	—	—	—	✓	✓
	Maintenance severity	—	—	✓	—	✓	✓	✓
	Normalized cyclomatic complexity	✓	✓	—	—	—	✓	✓
	Pathological complexity	—	—	—	—	—	—	✓
	Percent comments	—	—	✓	—	✓	✓	✓
Class attribute	Defective	✓	✓	✓	✓	✓	✓	✓

**Table 4:** Measurements to evaluate the experimental results.

S. No.	Measure	Equation
1	MAE	MAE=(1/2)∑_*j*=1_^*n*^|*y*_*i*_ − *y*|
2	RMSE	$\text{RMSE}=\;\sqrt{\left(1/2\right)\sum_{j=1}^{n}{\left(y_{i}-1\right)}^{2}}$
3	RAE	$\text{RAE}=\;\left(\left(\sum_{j=1}^{n}\left|P_{ij}-T\right|\right)/\left(\sum_{j=1}^{n}\left|T_{j-}\bar{T}\right|\right)\right)$
4	RRSE	$\text{RRSE}=\;\sqrt{\left(\left(\sum_{j=1}^{n}{\left(P_{ij}-T_{j}\right)}^{2}\right)/\left(\sum_{j=1}^{n}{\left(T_{j}-T\right)}^{2}\right)\right)}$
5	Recall	Recall=TP/(TP+FN)
6	Accuracy	Accuracy= (TP+TN)/(TP+TN+FP+FN)

**Table 5:** Comparative analysis of correctly classified instances.

S. No.	Technique	AR1	AR3	CM1	JM1	KC2	KC3	MC1
1	SVM	111	56	446	7842	432	159	9398
2	J48	109	55	438	7668	425	154	9406
3	RF	109	58	444	7930	435	158	9417
4	MLP	109	59	436	7863	442	150	9411
5	RBF	111	55	446	7869	437	155	9398
6	HMM	112	55	449	1759	415	36	9398
7	CDT	112	55	445	7833	433	159	9407
8	A1DE	110	58	430	7816	435	155	9297
9	NB	103	57	425	7810	436	153	8913
10	KNN	109	54	422	7395	420	140	9418

**Table 6:** Comparative analysis of incorrectly classified instances.

S. No.	Technique	AR1	AR3	CM1	JM1	KC2	KC3	MC1
1	SVM	10	7	52	1751	90	35	68
2	J48	12	8	60	1925	97	40	60
3	RF	12	5	54	1663	87	36	49
4	MLP	12	4	62	1730	80	44	55
5	RBF	10	8	52	1724	85	39	68
6	HMM	9	8	49	7834	107	158	68
7	CDT	9	8	53	1760	89	35	59
8	A1DE	11	5	68	1777	87	39	169
9	NB	18	6	73	1783	86	41	553
10	KNN	12	9	76	2198	102	54	48

**Table 7:** Comparative analysis of TPR and FPR of ML technique on different datasets.

Dataset		SVM	J48	RF	MLP	RBF	HMM	CDT	A1DE	NB	KNN
AR1	TPR	0.917	0.901	0.901	0.901	0.917	0.926	0.926	0.909	0.851	0.901
	FPR	0.926	0.723	0.928	0.723	0.926	0.926	0.926	0.927	0.523	0.621
AR3	TPR	0.889	0.873	0.921	0.937	0.873	0.873	0.873	0.921	0.905	0.857
	FPR	0.657	0.446	0.332	0.33	0.766	0.873	0.873	0.332	0.227	0.555
CM1	TPR	0.896	0.88	0.892	0.876	0.896	0.902	0.894	0.863	0.853	0.847
	FPR	0.902	0.849	0.848	0.886	0.902	0.902	0.902	0.869	0.616	0.762
JM1	TPR	0.817	0.799	0.827	0.82	0.82	0.183	0.817	0.815	0.814	0.771
	FPR	0.812	0.631	0.635	0.77	0.757	0.183	0.695	0.662	0.658	0.551
KC2	TPR	0.828	0.814	0.833	0.847	0.837	0.795	0.83	0.833	0.835	0.805
	FPR	0.634	0.422	0.431	0.435	0.472	0.795	0.439	0.424	0.473	0.432
KC3	TPR	0.82	0.794	0.814	0.773	0.799	0.186	0.82	0.789	0.789	0.722
	FPR	0.792	0.562	0.707	0.609	0.797	0.186	0.663	0.561	0.52	0.728
MC1	TPR	0.993	0.994	0.995	0.994	0.993	0.993	0.994	0.982	0.942	0.995
	FPR	0.993	0.701	0.657	0.73	0.993	0.993	0.774	0.628	0.38	0.496

**Table 8:** Comparative analysis of MAE.

S. No.	Technique	AR1	AR3	CM1	JM1	KC2	KC3	MC1
1	SVM	0.826	0.1111	**0.1044**	**0.1825**	**0.1724**	**0.1804**	**0.0072**
2	J48	0.127	0.1606	0.1757	0.2573	0.2374	0.2372	0.01
3	RF	0.127	0.1479	0.1631	0.2479	0.2205	0.257	0.0083
4	MLP	**0.1037**	0.1101	0.1568	0.2569	0.2259	0.2371	**0.0072**
5	RBF	0.1556	0.1812	0.1816	0.2773	0.2395	0.2995	0.025
6	HMM	0.5	0.5	0.5	0.5	0.5	0.5	0.5
7	CDT	0.1378	0.209	0.1745	0.2633	0.2296	0.2802	0.0112
8	A1DE	0.157	**0.105**	0.1886	0.2591	0.197	0.2708	0.0258
9	NB	0.1519	**0.1085**	0.1524	0.1863	**0.1638**	0.2162	0.059
10	KNN	0.1044	0.155	0.155	0.2319	0.2114	0.2809	**0.0063**

The bold values in the table indicate the reduced error rate.

**Table 9:** Comparative analysis of RAE.

S. No.	Technique	AR1	AR3	CM1	JM1	KC2	KC3	MC1
1	SVM	**57.249**	47.908	**58.379**	**60.9388**	52.7775	**59.2313**	49.9624
2	J48	87.9769	69.248	98.2132	85.9021	72.675	77.8877	69.4547
3	RF	87.9611	63.4368	91.1945	82.7532	67.4929	84.3792	57.6946
4	MLP	71.8266	47.4611	87.6482	85.7559	69.135	77.8521	49.9963
5	RBF	107.8175	78.1281	100.974	92.5753	73.3103	98.3279	174.0763
6	HMM	346.3562	215.586	279.5455	166.9291	153.0549	164.1553	3477.5284
7	CDT	95.4752	90.1037	97.5893	87.9121	70.29	91.9819	78.072
8	A1DE	108.7465	**43.7714**	105.4305	86.5138	60.3	88.8947	179.4312
9	NB	105.249	46.7686	85.2218	62.2139	**50.1471**	70.9899	410.217
10	KNN	72.3151	66.846	86.6364	77.4311	64.7095	92.209	**44.0253**

The bold values in the table indicate the reduced error rate.

**Table 10:** Comparative analysis of RMSE.

S. No.	Technique	AR1	AR3	CM1	JM1	KC2	KC3	MC1
1	SVM	0.2875	0.3333	0.3231	0.4272	0.4152	0.4247	0.0848
2	J48	0.2997	0.3424	0.3301	0.4053	0.3968	0.43	0.0779
3	RF	0.2856	0.2724	0.2951	**0.3577**	0.349	**0.3667**	**0.0669**
4	MLP	0.2882	**0.256**	0.3121	0.3706	0.3419	0.4414	0.0754
5	RBF	0.2664	0.2939	**0.2919**	0.3683	**0.3413**	0.3879	0.0837
6	HMM	0.5	0.5	0.5	0.5	0.5	0.5	0.5
7	CDT	**0.2627**	0.3377	0.3046	0.3752	0.3627	0.3818	0.0772
8	A1DE	0.2931	0.2925	0.3183	0.3754	0.3554	0.4034	0.1184
9	NB	0.3733	0.3176	0.38	0.4291	0.4019	0.4546	0.24
10	KNN	0.3122	0.3719	0.3905	0.475	0.4427	0.5246	0.0712

The bold values in the table indicate the reduced error rate.

**Table 11:** Comparative analysis of RRSE.

S. No.	Technique	AR1	AR3	CM1	JM1	KC2	KC3	MC1
1	SVM	109.405	99.6674	108.4851	110.4067	102.8529	109.2121	100.3607
2	J48	114.0496	102.3912	110.822	104.7491	98.2924	110.5573	92.2254
3	RF	108.6878	81.4368	99.0872	**92.4278**	86.4543	**94.2824**	**79.2174**
4	MLP	109.6657	**76.5306**	104.785	95.7816	84.6955	113.4827	89.3325
5	RBF	101.3862	87.8669	**97.9878**	95.1733	**84.5435**	99.7454	99.0846
6	HMM	190.2829	149.5011	167.8622	129.2111	123.8513	128.5606	592.0558
7	CDT	**99.9593**	100.9585	102.2522	96.9708	89.8344	98.1628	91.4393
8	A1DE	111.5568	87.4683	106.8639	97.0031	88.0436	103.724	140.1728
9	NB	142.0683	94.9565	127.572	110.8776	99.5502	116.8883	284.2012
10	KNN	118.7971	111.1859	131.084	122.7563	109.6576	134.8914	84.3477

The bold values in the table indicate the reduced error rate.

**Table 12:** Comparative analysis of recall.

S. No.	Technique	AR1	AR3	CM1	JM1	KC2	KC3	MC1
1	SVM	0.917	0.889	0.896	0.817	0.828	**0.82**	0.993
2	J48	0.901	0.873	0.88	0.799	0.814	0.794	0.994
3	RF	0.901	0.921	0.892	**0.827**	0.833	0.814	**0.995**
4	MLP	0.901	**0.937**	0.876	0.82	**0.847**	0.773	0.994
5	RBF	0.917	0.873	0.896	0.82	0.837	0.799	0.993
6	HMM	**0.926**	0.873	**0.902**	0.183	0.795	0.186	0.933
7	CDT	**0.926**	0.873	0.894	0.817	0.83	**0.82**	0.994
8	A1DE	0.909	0.921	0.863	0.815	0.833	0.799	0.982
9	NB	0.851	0.905	0.853	0.814	0.835	0.789	0.942
10	KNN	0.901	0.857	0.847	0.771	0.805	0.722	0.995

The bold values in the table indicate the highest recall in each column.

**Table 13:** The results of different techniques in terms of accuracy along with the rank values (it ranks the technique for each dataset separately, the best performing algorithm getting the rank of 1 and the second-best rank 2. Last two columns present the sum and average of ranks for each technique.).

	SVM	J48	RF	MLP	RBF	HMM	CDT	A1DE	NB	KNN
AR1	91.73 (2.5)	90.08 (4.25)	90.08 (4.25)	90.08 (4.25)	91.73 (2.5)	92.56 (1.5)	92.56 (1.5)	90.90 (3)	85.12 (5)	90.08 (4.25)
AR3	88.88 (5)	87.30 (6.33)	92.06 (3.5)	93.65 (2)	87.30 (6.33)	97.30 (1)	87.30 (6.33)	92.06 (3.5)	90.47 (4)	85.71 (7)
CM1	89.55 (2.5)	87.95 (5)	89.15 (4)	87.55 (6)	89.55 (2.5)	90.16 (1)	89.35 (3)	86.34 (7)	85.34 (8)	84.39 (9)
JM1	81.74 (4)	79.93 (8)	82.66 (1)	81.96 (3)	82.02 (2)	18.33 (10)	81.65 (5)	81.47 (6)	81.41 (7)	77.08 (9)
KC2	82.75 (6)	81.41 (7)	83.33 (4.5)	84.67 (1)	83.71 (2)	79.50 (9)	82.95 (5)	83.33 (4.5)	83.52 (3)	80.45 (8)
KC3	81.95 (1.5)	79.38 (4)	81.44 (2)	77.31 (7)	79.89 (3.5)	18.55 (9)	81.95 (1.5)	79.89 (3.5)	78.86 (6)	72.16 (8)
MC1	99.28 (5.33)	99.36 (4)	99.48 (1.5)	99.41 (2)	99.28 (5.33)	99.28 (5.33)	99.37 (3)	98.21 (6)	94.15 (7)	99.49 (1.5)
Sum (accuracy)	615.93	605.43	618.23	614.66	613.52	495.70	615.16	612.24	598.90	589.39
Average (accuracy)	87.99	86.49	88.32	87.81	87.65	70.81	87.88	87.46	85.56	84.20
Sum (rank)	26.83	38.58	20.75	25.25	24.16	36.83	25.33	33.50	40.00	46.75
Average (rank)	3.83	5.51	2.96	3.61	3.45	5.26	3.62	4.79	5.71	6.68

**Table 14:** Decision table.

Datasets	Evaluation measures					
	MAE	RAE	RMSE	RRSE	Recall	Accuracy
AR1	MLP	SVM	CDT	CDT	HMM, CDT	HMM, CDT
AR3	A1DE, NB	A1DE	MLP	MLP	MLP	HMM
CM1	SVM	SVM	RBF	RBF	HMM	HMM
JM1	SVM	SVM	RF	RF	RF	RF
KC2	NB, SVM	NB	RBF	RBF	MLP	MLP
KC3	SVM	SVM	RF	RF	SVM	SVM
MC1	KNN, SVM, MLP	KNN	RF	RF	RF	KNN, RF

**Table 15:** Family of hypotheses ordered by the *P* value and adjusting *α* by Nemenyi and Holm's procedures, considering an initial *α* = 0.05.

S. No.	Algo versus algo		*z*	*P*	NM (0.05)	Holm	*R*_*i*_ − *R*_*j*_	CD
1	RF	KNN	14.8740	6.07*E* − 08	0.001	0.0011	3.7143	>
2	RBF	KNN	12.9232	2.04*E* − 07	0.001	0.0011	3.2271	>
3	MLP	KNN	12.2997	3.12*E* − 07	0.001	0.0012	3.0714	>
4	CDT	KNN	12.2539	3.22*E* − 07	0.001	0.0012	3.0600	>
5	SVM	KNN	11.3958	5.97*E* − 07	0.001	0.0012	2.8457	>
6	RF	NB	11.0125	7.97*E* − 07	0.001	0.0013	2.7500	>
7	J48	RF	10.2001	1.52*E* − 06	0.001	0.0013	2.5471	>
8	RF	HMM	9.1990	3.57*E* − 06	0.001	0.0013	2.2971	>
9	RBF	NB	9.0617	4.04*E* − 06	0.001	0.0014	2.2629	>
10	MLP	NB	8.4381	7.21*E* − 06	0.001	0.0014	2.1071	>
11	CDT	NB	8.3924	7.53*E* − 06	0.001	0.0014	2.0957	>
12	J48	RBF	8.2494	8.65*E* − 06	0.001	0.0015	2.0600	>
13	J48	MLP	7.6258	1.62*E* − 05	0.001	0.0015	1.9043	>
14	J48	CDT	7.5800	1.7*E* − 05	0.001	0.0016	1.8929	>
15	A1DE	KNN	7.5800	1.7*E* − 05	0.001	0.0016	1.8929	>
16	SVM	NB	7.5343	1.78*E* − 05	0.001	0.0017	1.8814	>
17	RF	A1DE	7.2940	2.3*E* − 05	0.001	0.0017	1.8214	>
18	RBF	HMM	7.2482	2.41*E* − 05	0.001	0.0018	1.8100	>
19	SVM	J48	6.7219	4.32*E* − 05	0.001	0.0019	1.6786	>
20	MLP	HMM	6.6247	4.83*E* − 05	0.001	0.0019	1.6543	>
21	HMM	CDT	6.5789	5.09*E* − 05	0.001	0.0020	1.6429	>
22	SVM	HMM	5.7208	0.000143	0.001	0.0021	1.4286	>
23	HMM	KNN	5.6750	0.000152	0.001	0.0022	1.4171	>
24	RBF	A1DE	5.3432	0.000233	0.001	0.0023	1.3343	>
25	MLP	A1DE	4.7196	0.000545	0.001	0.0024	1.1786	>
26	J48	KNN	4.6739	0.000581	0.001	0.0025	1.1671	>
27	CDT	A1DE	4.6739	0.000581	0.001	0.0026	1.1671	>
28	NB	KNN	3.8615	0.001919	0.001	0.0028	0.9643	>
29	SVM	A1DE	3.8158	0.002058	0.001	0.0029	0.9529	>
30	A1DE	NB	3.7185	0.002391	0.001	0.0031	0.9286	>
31	SVM	RF	3.4782	0.003479	0.001	0.0033	0.8686	>
32	J48	A1DE	2.9062	0.00871	0.001	0.0036	0.7257	>
33	RF	CDT	2.6201	0.013903	0.001	0.0038	0.6543	<
34	RF	MLP	2.5743	0.014987	0.001	0.0042	0.6429	<
35	RF	RBF	1.9508	0.041431	0.001	0.0045	0.4871	<
36	HMM	A1DE	1.9050	0.044585	0.001	0.0050	0.4757	<
37	HMM	NB	1.8135	0.051582	0.001	0.0056	0.4529	<
38	SVM	RBF	1.5274	0.080499	0.001	0.0063	0.3814	<
39	J48	HMM	1.0011	0.171458	0.001	0.0071	0.2500	<
40	SVM	MLP	0.9039	0.194805	0.001	0.0083	0.2257	<
41	SVM	CDT	0.8581	0.206548	0.001	0.0100	0.2143	<
42	J48	NB	0.8124	0.218775	0.001	0.0125	0.2029	<
43	RBF	CDT	0.6693	0.260042	0.001	0.0167	0.1671	<
44	MLP	RBF	0.6236	0.274195	0.001	0.0250	0.1557	<
45	MLP	CDT	0.0458	0.482248	0.001	0.0500	0.0114	<

## Data Availability

The datasets used in this research are taken from UCI ML Learning Repository available at https://archive.ics.uci.edu/.
